This article has been retracted.

# Study on Syndrome Intervention of Nonalcoholic Fatty Liver Disease from the Perspective of Deficiency and Excess

**DOI:** 10.1155/2021/9928160

**Published:** 2021-09-15

**Authors:** Sanhang Wang, Hu Jiu lüe, Jiao Zhao

**Affiliations:** Zhang Zhongjing School of TCM, Nanyang Institute of Technology, Nanyang 473004, Henan, China

## Abstract

During the onset of nonalcoholic fatty liver disease (NAFLD), the original deficiency is the root cause of its occurrence, and the actual condition is the basic condition for its occurrence. Therefore, the correlation between the deficiency and the actual condition is the basic law of NAFL syndrome formation, pathogenesis, development, and change. Based on this, the purpose of this article is to study and analyze the syndrome intervention of NAFLD from the perspective of the original deficiency and the true standard. In this article, the TCM physical fitness determination and related risk factors investigation were conducted on qualified NAFLD patients collected from outpatient clinics and physical examination centers of a certain local hospital. Analyze the correlation between the physique bias, physique type, and risk factors of NAFLD patients, in order to effectively carry out Chinese medicine “preventive treatment” in the future. Predicting the risk of nonalcoholic fatty liver disease from the perspective of physique, more targeted health education for NAFLD patients with risk factors, reducing the risk of nonalcoholic fatty liver disease, and providing evidence for prevention and treatment of fatty liver. The research in this article aims to show a clearer conclusion on the structural characteristics of NAFLD's syndromes related to the deficiency of the original standard and the actual syndromes or the syndromes related to the original deficiency of the standard of the actual syndromes; NAFLD has the characteristics of being related to the original deficiency and the actual standard, and the relationship between the original deficiency and the actual standard has different syndromes, and the relationship between the original deficiency and the actual standard can also show the characteristics of different subsyndromes. Experimental research shows that people with hot and humid constitution are prone to suffer from hyperglycemia, intermediate coke hot and heat obstruction, spleen and stomach clearance, and turbidity reduction function is impaired, and the migration and transformation of water and valley essence after the stomach is uneven, leading to the stagnation of water, wet, phlegm, blood stasis, and other pathological products.

## 1. Introduction

The research of nonalcoholic fatty liver disease is still in the exploratory stage in traditional Chinese medicine, including the name of the disease and the classification of syndromes in traditional Chinese medicine have not yet been unified, and the treatment needs to be standardized. In the process of its onset, the original deficiency is the root cause of its occurrence, and the standard reality is the basic condition for its occurrence [1, 2].

There are also many personal experience prescriptions for the treatment of NAFLD. For example, Chen Xie et al. believe that there are more turbid phlegm in obese NAFLD patients, so products that invigorate the spleen, eliminate phlegm, and remove dampness can be reused in treatment, such as *Poria*, *Coix* seed, and *Alisma*. People with high blood pressure and diabetes often have mutual obstruction of phlegm and blood stasis and also suffer from NAFLD. The treatment principle is recommended to promote blood circulation to remove blood stasis, dredge collaterals, and remove dampness. Commonly used drugs include vinegar Bupleurum, Wulingzhi, peach kernel, and Danshen; in patients with NAFLD and frail elderly, weakness of spleen Qi and loss of the liver and kidney often occur. The treatment principle is to invigorate the spleen and replenish Qi, liver, and kidney. Commonly used drugs include *Rhodiola*, *Astragalus*, fleece-flower root, and Rehmannia glutinosa [3].

This experiment collected data from patients in a certain place to investigate the body mass index and fasting glucose. In order to ensure the scientific nature and comprehensiveness of the experiment, it is grouped according to the physiological situation of patients. The patients were divided into normal body mass index and high group and fasting normal blood glucose group and high blood sugar group. On this basis, the subject of this article is researched and analyzed through the experimental comparison and analysis.

## 2. Discuss the Research of NAFLD's Syndrome Intervention Treatment from the Perspective of the Deficiency of the Essence and the Essence

### 2.1. NAFLD Etiology and Pathogenesis

#### 2.1.1. Irregular Diet

“Suwen's Different Formula Theory” states that “accumulation” and “gas” patients tend to have rich clothing and food. Eating is too good and is less affected by external evils. Most of the disease comes from the internal growth of sputum in the human body. Generally, people who adhere to the principle of “food and essence nutrition” are more likely to appear endogenous phlegm dampness, leading to phlegm dampness blocking the spleen and stomach, spleen and stomach gas congestion, bilateral phlegm dampness and blood stasis, leading to NAFLD. In ancient times, people's living standards were generally low. After all, there were a few people who had good food and clothing. The general population suffering from “hypochondriac pain” may be related to hunger and fullness and irregular diet [4, 5]. In short, most doctors agree that the onset of the fatty liver is inseparable from irregular eating time, uncontrollable drinking, excessive consumption of fried and greasy food, long-term sitting in front of the computer, and lack of exercise, which makes the spleen lose movement and cannot transform water and grains. The elderly chronically ill, combined with insufficient kidney essence and powerlessness, can cause phlegm dampness and blood stasis to condense in the liver. Chinese medicine also recognizes that causal circulation, phlegm, and stasis are both pathological products, which in turn can lead to the further development of the disease [6, 7].

#### 2.1.2. Emotional Disorders

The liver was called the officer of the generals by ancient Chinese medicine, with sexual pleasure and depression [8, 9]. The most important function of the liver is summarized as the liver governs venting. If emotional depression or irritability, these symptoms accumulate in the liver and cause hypochondriac pain, hypochondriac swelling, and other manifestations; clinical findings show that patients with hypochondriac pain are more depressed and unhappy, or impatient anger is about the dysfunction of military officials and the inability of liver Qi to drain normally, leading to the fatty liver [10, 11].

#### 2.1.3. Loss of Work and Rest

Overwork depletes vitality, and Qi plays a role in promoting body fluid movement in the body [12]. If the body fluid is not running smoothly, it will cause various diseases including the nonalcoholic fatty liver. The limbs are dominated by the spleen, and the Qi and blood flow is stagnant, which in turn affects the spleen's transportation and transformation functions, causing the spleen to lose health, phlegm, and dampness obstructed by the liver, and the pulse is the disease; or because of the rapid pace of life and excessive work pressure too much, staying up late, and working overtime too frequently, the liver and blood are drained. At the same time, the essence of the kidney is the foundation of the whole body, which is related to the body's internal organs. Kidney deficiency and spleen will eventually become phlegm and blood stasis.

#### 2.1.4. Physical Reasons

The clinical application of constitution theory research on NAFLD found that phlegm dampness traps the spleen, which affects the movement and transformation of the spleen and stomach; the spleen and stomach are the lifting and lowering hub of the Qi machine, and the liver Qi depends on the flow of the Qi machine. The “Secret Record of the Stone Chamber” once said that fat people have a lot of phlegm in their bodies. This is due to the deficiency of vital energy, which cannot carry body fluid, so phlegm is produced. Qi deficiency affects the up and down of the spleen and stomach, the dampness stays, the dampness accumulates into phlegm, the dampness of phlegm drink is easy to become stagnant and heat, and dampness and heat fight each other, resulting in the fatty liver. Therefore, people with phlegm dampness, Qi deficiency, and damp-heat are susceptible to the fatty liver.

### 2.2. Empirical Analysis of NAFLD's False Standard

#### 2.2.1. The Structural Characteristics and Change Characteristics of NAFLD's Empirical Syndrome

The so-called NAFLD main deficiency syndrome refers to the pathological state that NAFLD syndrome manifests in the development and change process of the evil, and the positive and the deficiency is the root cause of the disease, and the evil is the basic condition of the disease. NAFLD is manifested in the characteristics of the positive syndromes of the original deficiency standard, or the deficiency in the actual, or the deficiency in the deficiency, or the interlacing of the deficiency and the actual, or the combination of the deficiency and the actual syndrome, how the deficiency and the reality are related, and the specific syndromes related to the deficiency, and the actual types of NAFLD have not been elaborated in the previous textbooks and reference materials. Therefore, further in-depth research is needed. In any case, the clinical manifestations of NAFLD's primary deficiency syndromes and subsyndrome related to primary deficiency syndromes and real syndromes should be based on the main syndrome manifestation categories with primary syndromes related to primary deficiency syndromes. Therefore, the focus of this research is to first establish the standard syndrome database of NAFL's original syndrome of deficiency of the original syndrome and the subsyndrome related to the original deficiency of the syndrome.

#### 2.2.2. The Evolution Law of the Syndromes Related to NAFLD's Original Deficiency and Standard Excess

Any syndrome change has its own characteristics and laws. The development and changes of NAFLD's syndromes related to the deficiency of the original syndrome and the syndromes related to the deficiency of the original syndrome and the subsyndromes of the original syndrome must also have certain characteristics and rules. Through the in-depth special research of this project, patients undergo retrospective clinical follow-up; follow the patients at a set time period and intervene with Ganzhiping capsule drugs, aiming to reveal the types of syndromes related to the deficiency of NAFLD and the changes in the subsyndrome structure of the syndromes related to the deficiency of NAFLD. Combined with the preliminary research we conducted, we should be able to discover the inherent laws of the development and evolution of the syndrome types related to the deficiency of the original deficiency and the excess of the standard and the development and evolution of the syndromes related to the deficiency and the excess of the original syndrome.

### 2.3. Analysis of TCM Syndromes and Clinical Features of NAFLD

#### 2.3.1. The Composition of Various Syndrome Types in TCM Dialectics

A total of 69 cases of internal medicine in a hospital in a certain area were included in this study, and the specific distribution is shown in Figure 1.

Analyzed from the composition of the number of cases, the number of patients with phlegm and blood stasis obstructing collaterals is the most and the number of patients with kidney deficiency is the least. Previous studies have found that the pathogenesis of nonalcoholic fatty liver disease is mainly responsible for pathological factors such as phlegm, blood stasis, dampness, and turbidity in the etiology of Chinese medicine. According to the analysis of syndrome differentiation, the pathogenesis characteristics of the cases included in this study are actual or deficient, as well as mixed with deficient and actual symptoms. The syndrome of phlegm and blood stasis obstructs the collaterals if the pathogenesis is true.

#### 2.3.2. Frequency of Use of Traditional Chinese Medicine

Analyze the frequency of use of each medicine according to the following formula:

(1) $$\begin{array}{c} Fi=\frac{Ni}{M}. \end{array}$$

Among them, *Fi* is the frequency of use of the *i*^th^ Chinese medicine (%), and *Ni* is the frequency of use of the *i*^th^ Chinese medicine. After research and analysis, a total of 11 medicines have a frequency of use greater than 1, as shown in Figure 2.

In clinical research, “testing syndromes with prescriptions” is one of the commonly used methods of contradiction. In this study, the analysis results from the drug point of view are basically consistent with the clinical data analysis results.

#### 2.3.3. Analysis of medication classification

The proportion of each type of medicine is calculated according to the following formula:

(2) $$\begin{array}{c} Pi=\frac{Ni}{M}, \end{array}$$

where *Pi* is the proportion (%) of type *i* Chinese medicine used, and *Ni* is the number of times that type *i* Chinese medicine is used. The details are given in Table 1.

## 3. Exploring the Experimental Study of the Nonalcoholic Fatty Liver from the Point of View of Deficiency and Excess

### 3.1. Research Objects

Select 300 NAFLD patients from a certain place as the research object.

### 3.2. Inclusion Criteria

1. Patients in the healthcare department and physical examination center who meet the criteria of nonalcoholic fatty liver disease diagnosed by Western medicine are 18–65 years old
2. The case data are complete and reliable, and those who agree to the investigation.

### 3.3. Exclusion Criteria

1. Patients found to have alcoholic fatty liver and drug-induced liver disease after examination
2. The information is incomplete and does not agree with the investigation

### 3.4. Research Methods

#### 3.4.1. Comparative Method

Combined with the actual situation of this survey, the body mass index and other comparative studies were carried out to analyze the research content of this article.

#### 3.4.2. Cross-Sectional Survey Method

Based on the informed consent of the survey subjects, the TCM physicians from the healthcare department and the prevention center will carry out on-site investigations and related project inspections to obtain the population's TCM physique distribution, collect risk factor data, and determine risk factor groups. Finally, the monkey hurriedly collected and sorted out and concluded.

#### 3.4.3. Mathematical Statistics

Use related software to conduct split statistics on the research results of this article.

## 4. Exploring the Experimental Analysis of the Nonalcoholic Fatty Liver from the Perspective of the Deficiency and the Excess

### 4.1. Distribution of Tcm Physique Types of NAFLD Patients with Different Body Mass Indexes

According to the criteria for Asians proposed by the WHO Western Pacific Region Obesity Task Force, 300 NAFLD patients were divided into two groups: normal weight and overweight. The data obtained are given in Table 2.

According to Figure 3, the physical distribution of 300 NAFLD patients is the most phlegm and wet, followed by humid heat, gas deficiency, blood stasis, Yang deficiency, Yin deficiency, gas stagnation, and other characteristics. The investigation made no findings (Table 3).

It can be seen from Figure 4 that the type of physique is correlated with abnormal blood glucose. This study found that people with damp and hot constitution are prone to high blood sugar. Patients with high blood sugar usually prefer sweet and greasy products, which tend to cause dampness and heat to accumulate, the spleen likes dryness and disgusting dampness, the spleen becomes healthy, and the stomach Qi becomes peaceful. Patients with damp-heat type tend to have weak spleen and stomach. Due to damp-heat obstruction of the middle coke, the function of the spleen and stomach to raise clearing and reduce turbidity is impaired and causes pathological products such as watery dampness, phlegm, and blood stasis to remain in the blood vessels and collaterals, and phlegm and blood stasis are mutually agglomerated in the liver over time, forming the fatty liver.

## 5. Conclusion

In the prevention and control of NAFLD, the Chinese medicine has a unique advantage. As early as the Huang Di era more than 5,000 years ago, people believed that the most intelligent doctor could see the clues before the disease occurred and take timely measures to treat the disease. The story of Bian Que's meeting with Cai Huangong demonstrates the importance of prevention. It may be too late to treat the disease until it occurs. Doctors can only stand in a passive position. TCM emphasizes “adjusting measures according to individual circumstances.” In fact, adaptation measures under individual conditions are also based on physical conditions. Study the relationship between the risk factors of NAFLD and the constitution of traditional Chinese medicine from the physical perspective, reduce the risk of fatty liver disease, focus on improving the risk awareness of fatty liver sensitive patients, regulate the diet, exercise, work, rest, and spirit, make the pathological physique into a calm physique, and finally reduce the risk of pain.

## Figures and Tables

**Figure 1:** Gender composition of TCM syndromes in each group.

**Figure 2:** Drugs used more than 1%.

**Figure 3:** Distribution of BMI and TCM physique types of NAFLD patients.

**Figure 4:** The distribution of blood glucose and physical fitness in patients with NAFLD.

**Table 1:** The proportion and frequency of use of various types of traditional Chinese medicine.

	Use ratio	Usage frequency
Nourishing Qi and spleen medicine	7.69	22.38
Activating blood and removing blood stasis medicine	5.13	14.70
Qi regulating medicine	3.85	12.81
Aromatic wet medicine	3.85	8.35
Diuresis and dampness medicine	3.21	7.24
Resuscitation medicine	2.56	5.46
Laxative	2.56	4.45

**Table 2:** Distribution of BMI and TCM physique types of NAFLD patients.

	BMI normal group	BMI abnormal group
Phlegm quality	20	103
Heat and humidity	20	28
Qi deficiency	18	24
Blood stasis	14	19
Yang deficiency	9	12
Yin deficiency	7	10
Peace	3	3
Temperament	4	6
Idiosyncratic	0	0

**Table 3:** The distribution of blood glucose and physical fitness in patients with NAFLD.

	Normal blood sugar group	Abnormal blood sugar group
Phlegm quality	60	68
Heat and humidity	10	38
Qi deficiency	20	22
Blood stasis	15	18
Yang deficiency	8	9
Yin deficiency	10	11
Peace	3	3
Temperament	4	6
Idiosyncratic	0	0

## Data Availability

The data used to support the findings of this study are included within the article.
